The article "Artificial Intelligence Auxiliary Algorithm for Wushu Routine Competition Decision Based on Feature Fusion" was retracted in 2023. Reasons: signs of a paper mill; suspected computer-generated content; unreliable results or conclusions; concerns about the data.

# Artificial Intelligence Auxiliary Algorithm for Wushu Routine Competition Decision Based on Feature Fusion

**DOI:** 10.1155/2021/1632393

**Published:** 2021-08-11

**Authors:** Chao Zhao, Bing Li

**Affiliations:** ^1^Wushu College WuHan Sports University, Wuhan 430079, Hubei, China; ^2^Yong in Univerity Korea, Cheoin-gu, Yongin-si, Gyeonggi-do 17092, Republic of Korea

## Abstract

The developments of modern science and technology have significantly promoted the progress of sports science. Advanced technological methods have been widely used in sports training, which has not only improved the scientific level of training but also promoted the continuous growth of sports technology and competition results. Competitive Wushu routine is an important part of Chinese Wushu. The development trend of competitive Wushu routine affects the development of the whole Wushu movement. To improve the training effect of the Wushu routine using artificial intelligence, this paper employed fuzzy information processing and feature extraction technology to analyze the visual features in the process of Wushu competition. The deep neural network-based region segmentation method was employed for implicit feature extraction to examine the shape, texture, and other image features of Wushu routines and improve the recognition performance. The proposed feature extraction model achieved the highest average accuracy of 93.98% accuracy as compared to other contemporary algorithms. Finally, the model was evaluated to validate the superior performance of the proposed method in improving the decision-making ability and effective instruction ability of the martial arts routine competition.

## 1. Introduction

Wushu, formed gradually in the course of historical development, is a kind of integration of multiethnic cultures and the common cultural wealth of mankind [1]. It contains rich contents, including cultural, economic [2], religious, and political and is the organic combination of culture, sports, and art. Standing at the historical starting point of the new era, all ethnic regions will continue to promote the comprehensive and coordinated development of traditional ethnic sports, mass sports [3], and competitive sports [4, 5], to make ethnic sports become an important guarantee for inspiring national spirit and increasing progress and development. Chinese martial arts have become the most influential and representative cultural standard symbol of Chinese culture and are also one of the traditional cultural characteristics of Chinese national sports. As an important part of Wushu, the development of competitive Wushu affects the development of Wushu to a great extent.

The appearance of the competitive Wushu routine [6, 7] is the product of history and the development of The Times. Chinese Wushu has been separated and formed several interrelated but different characteristic items, such as modern competitive Wushu and traditional Wushu. Competitive Wushu reflects and follows the characteristics and principles of competitive sports, such as the strict implementation of quantitative evaluation, and there are more refined scoring standards. As the “traditional Wushu” among the sports, it has been marked with the brand of competition since modern times, which also speeds up the transformation of the traditional Wushu into the competitive style and conforms to the historical situation and trend, which is worthy of the affirmation of the Chinese nation [8].

The article "Artificial Intelligence Auxiliary Algorithm for Wushu Routine Competition Decision Based on Feature Fusion" was retracted in 2023. Reasons: signs of a paper mill; suspected computer-generated content; unreliable results or conclusions; concerns about the data.

At present, Chinese Wushu has not been included in the Olympic Games [9], and the reasons mainly include many types of Wushu, difficulty in determining the event, and the difficulty in scoring the competition. But even if Wushu is not included in the Olympic Games, its profound cultural heritage and accumulation always show its exuberant vitality. The development of martial arts cannot only strengthen the body and enhance the national quality, but also is a kind of inheritance of China's nonmaterial civilization and can even form a new industrial form [10]. Currently, Chinese athletics martial arts career development is still faced with many problems such as lack of education of Wushu athletics, Wushu dissemination surface, and loss of Wushu skills [10]. From this perspective, the development of the new age of competitive Wushu is the dire need of new macroscopic development measures.

In the context of the continuous development of society, people's ability to control society has been significantly improved, and competitive martial arts and Wushu have a broader space for development. The research on the macro development of competitive Wushu routine is more concentrated than that of Wushu one-way sports [11, 12]. Therefore, the research focus is mostly on the generation and development of competitive Wushu routine, and to a large extent, it imitates the management mode of Western sports. Researchers focus on the analysis of the thoughts and intentions of the participants of competitive Wushu routine and focus on the exploration of the crowd of competitive Wushu routine, the ontology of competitive Wushu routine, and the extension of interests, but do not fully consider the perspective and integrity of the macrodevelopment of competitive Wushu routine, including the macrodevelopment path of competitive Wushu routine. The lack of research in this aspect makes it difficult for competitive Wushu routines to better adapt to the development of society, and it is urgent to change them with the development of The Times. The major contributions of this paper are as follows:

- This paper proposed a novel artificial intelligence-aided algorithm for Wushu routine competition decision-making based on feature fusion
- The paper proposed a deep neural network region segmentation method for implicit feature extraction to analyze the shape, texture, and other image features of martial arts routines which can effectively improve the recognition performance of martial arts routines.

The article "Artificial Intelligence Auxiliary Algorithm for Wushu Routine Competition Decision Based on Feature Fusion" was retracted in 2023. Reasons: signs of a paper mill; suspected computer-generated content; unreliable results or conclusions; concerns about the data.

The rest of this paper is organized as follows.  Section 2 discusses the related work in martial arts competitions followed by the methodology section. The experimental results are presented in Section 4. Finally, Section 5 concludes the paper with summary and future research directions.

## 2. Related Work

### 2.1. Competitive Martial Arts Routines

Since the 1950s, competitive Wushu has gradually formed and developed based on traditional Wushu. Competitive Wushu is a modern competitive sport in China that is based on the rules of competition with routine and free Shushu as the two main activities. The competitive Wushu routine is formed after the integration of Chinese and Western sports culture which belongs to the modernization of Wushu. Scholars define the concept of “competitive Wushu” with respect to the formation, evolution, and development of the competitive Wushu routine [13].

To reflect the changes in Wushu routines, athletes should have good strength, speed, agility, and flexibility. The extraction of images for different actions can effectively judge the completion quality of Wushu actions. To study the difficult images of Wushu, it is necessary to extract the prominent features of different Wushu images.

With the rapid development of machine image recognition technology, the identification of Wushu actions has moved from an original method of artificial representation to advanced deep learning methods. Recently, with the expansion of video behavior and action recognition algorithms [14], it can be divided into two categories according to the types of the extracted action features, i.e., methods based on shallow features and deep learning [15].

A convolutional neural network (CNN) is a variant of deep learning algorithms and has a good expression of the two-dimensional features of the image. It can effectively combine the features of the previous moment to ensure that the network can understand the timing information. Since the video behavior can be viewed as a set of constant image sequences, a dual-stream network model architecture of CNN [16–18] combined with LSTM was developed. The main idea was to use the CNN to extract the three-dimensional characteristics of the video frame image, to capture the timing information between actions through the RNN network, and to collect the temporal and three-dimensional features [17] for the identification of actions in the video. In addition, the movement of the human body can be described by the movement of the skeleton joint points. Hence, a dual-stream RNN was used for spatial position and time dynamic characteristics of the human skeleton joint points for modeling, i.e., RNN-based methods [19] can directly pass Wushu video frames as input to the network to realize an end-to-end action recognition. This paper focuses on one application of video feedback system in the analysis and diagnosis of the Wushu routine movement and discusses its future development trend.

The article "Artificial Intelligence Auxiliary Algorithm for Wushu Routine Competition Decision Based on Feature Fusion" was retracted in 2023. Reasons: signs of a paper mill; suspected computer-generated content; unreliable results or conclusions; concerns about the data.

### 2.2. Preprocessing of Video Image of Wushu Routine Competition

The first step in the video processing [18] of the Wushu competition is the preprocessing of the images. Due to miscellaneous environmental factors such as the change of shooting position, light intensity, and shaking of the handheld camera, the collected video is mixed with different degrees of interference and noise which affects the image recognition accuracy. In the image process, the basic noise of the target image is eliminated and filters are applied to improve the image quality. The preprocessing of an image is further complicated by fading and incompleteness of the recorded video. To minimize the interference that affects the final processing result of the kernel algorithm, it is necessary to preprocess the image first. The quality of the image preprocessing technique has a great influence on subsequent [13, 20] targeted image tracking. This article mainly adopts the grayscale processing method. Its main function is to minimize background noise and enhance detection and tracking. Image preprocessing can reduce interference factors and improve the accuracy of target detection.  Figure 1 shows different images after preprocessing technique has been applied.

Gray image with basic color is white and black. Each image's brightness ranges from zero to hundred percent. Mostly, the color images are represented in the RGB model. If *R* = *G* = *B*, then color represents a grayscale color with a grayscale range of 0–255. Pixel in grayscale image stores brightness value in bytes, that is, grayscale value, one pixel corresponds to one byte. In the color image, the gray values of three gray images are used to express the brightness of the three components, and one gray image can be selected.

(1) $$\begin{array}{c} f_{1}\left(i,j\right)=R\left(i,j\right),\\ f_{2}\left(i,j\right)=G\left(i,j\right),\\ f_{3}\left(i,j\right)=B\left(i,j\right), \end{array}$$

where *f*_*k*_(*i*, *j*)(*k*=1,2,3) is the gray value of the converted gray image at (*i*, *j*). The following equation represents the grayscale image after the weighted average of the three components of RGB:

(2) $$\begin{array}{c} f\left(i,j\right)=0.30R\left(i,j\right)+0.59G\left(i,j\right)+0.11B\left(i,j\right). \end{array}$$

The article "Artificial Intelligence Auxiliary Algorithm for Wushu Routine Competition Decision Based on Feature Fusion" was retracted in 2023. Reasons: signs of a paper mill; suspected computer-generated content; unreliable results or conclusions; concerns about the data.

## 3. Methodology

### 3.1. Image Sampling of Martial Arts Routine Competition

To achieve the Wushu movement visual image recognition based on feature extraction, the Wushu movement region segmentation method is applied using frame section scanning techniques, and a visual feature reconstruction model is developed. Assuming that Wushu movement visual image grayscale pixel sets are P(*i*, *j*), routine action image characteristics such as shape, texture, and image gray value of *I*_swk_, the dataset to get the corresponding Wushu movement characteristics of visual components can be represented as

(3) $$\begin{array}{c} {\text{TC}}_{\text{rk}}=\left(\frac{\sum_{j=1}^{c}I_{\text{swk}}\left(1,j\right)}{c},\frac{\sum_{j=1}^{c}I_{\text{swk}}\left(2,j\right)}{c},\frac{\sum_{j=1}^{c}I_{\text{swk}}\left(i,j\right)}{c},\ldots ,\frac{\sum_{j=1}^{c}I_{\text{swk}}\left(r,j\right)}{c}\right),\\ {\text{TC}}_{\text{ck}}=\left(\frac{\sum_{j=1}^{c}I_{\text{swk}}\left(i,1\right)}{r},\frac{\sum_{j=1}^{c}I_{\text{swk}}\left(i,2\right)}{r},\frac{\sum_{j=1}^{c}I_{\text{swk}}\left(i,j\right)}{r},\ldots ,\frac{\sum_{j=1}^{c}I_{\text{swk}}\left(i,c\right)}{r}\right), \end{array}$$

where *c* is the column number of the visual feature of martial arts routines and *r* is the three-dimensional points on the motion model. Combined with the two-dimensional color image reconstruction method, the distribution characteristic quantity of martial arts routine action visual pixel set was obtained. The visual image of martial arts routine action was processed using fuzzy fusion, and the action visual tracking [21] and recognition were carried out. The dynamic analysis model of martial arts routine action features was constructed by image segmentation method, and the dynamic characteristic quantity was obtained:

(4) $$\begin{array}{c} G_{j}\left(\overset{⟶}{x}\right)=\left\{\begin{array}{cc} \max\left[0,g_{j}\left(\overset{⟶}{x}\right)\right], & 1\leq j\leq l,\\ \max\left[0,\left[h_{j}\left(\overset{⟶}{x}\right)-\delta \right]\right], & l+1\leq j\leq p. \end{array}\right) \end{array}$$

### 3.2. Feature Extraction of Wushu Routine Action

The edge feature segmentation method was employed to express and process the visual features of the Wushu Sanda whip movement, and the edge contour feature analysis model was developed. The edge feature extraction is used to isolate or extract the features of an object. Once the edges have been identified, we can analyze the image and identify the object. The visual distribution function of Wushu Sanda whip movement was calculated as

(5) $$\begin{array}{c} g=k⊗f+n, \end{array}$$

where ⊗ represents the morphological filter operator. The collected visual images of Wushu Sanda whip leg movement are fused and processed and the connected distribution set of features was computed as

(6) $$\begin{array}{c} S\left(t\right)=\sum_{i=0}^{i}\sum_{j=0}^{N_{p}-1}p\left(t-iT_{s}-jT_{p}-c_{j}T_{c}-a_{i}\varepsilon \right), \end{array}$$

where *T*_*s*_ is the location feature of the edge of the region. The watershed image segmentation algorithm is used to reconstruct the action of martial arts routines, and the dynamic feature decomposition model was established as follows:

(7) $$\begin{array}{c} x\left(t\right)=\sum_{m=0}^{M}\sum_{k=1}^{K\left(m\right)}w_{nk}s\left(t-T_{m}-\tau_{mk}\right)+v\left(t\right), \end{array}$$

where *w*_*mk*_ is the edge feature component of the martial arts routine. Using mathematical morphology, the three-dimensional modal output of the visual reconstruction of the martial arts routine is obtained as

(8) $$\begin{array}{c} \left\{\begin{array}{c} x=R\;\sin\;\eta \;\cos\;\phi ,\\ y=R\;\sin\;\eta \;\sin\;\phi ,\\ z=R\;\cos\;\eta . \end{array}\right) \end{array}$$

The article "Artificial Intelligence Auxiliary Algorithm for Wushu Routine Competition Decision Based on Feature Fusion" was retracted in 2023. Reasons: signs of a paper mill; suspected computer-generated content; unreliable results or conclusions; concerns about the data.

### 3.3. Martial Arts Routine Action Recognition and Assistant Decision Model

This section establishes an artificial intelligence [22–25] auxiliary algorithm for Wushu routine competition decision-making based on feature fusion.  Figure 2 shows the framework of the proposed martial arts routine recognition model. Initially, the collected Wush images are preprocessed to eliminate background noise and interference. Then, multifeature extraction methods [26–28] are applied to extract discriminant feature patterns from the preprocessed images. The extracted feature patterns are fused and provided as input to the proposed CNN model. The CNN model with multiple hidden layers was used to recognize routine actions and assist the data analysis team and coach team to make decisions.

## 4. Experiments and Results

### 4.1. Experimental Setup

To test the application performance of this method in realizing the visual image recognition of martial arts routine movements, the simulation experiment analysis was carried out using Matlab 7. The experimental parameters are shown in Table 1.

### 4.2. Dataset

The dataset used in this experiment was downloaded from the Internet. The dataset is comprised of a total of 8000 visual pictures of martial arts routines. From the given dataset, the low-quality images were eliminated and the high-quality 1700 images were selected for training the proposed model. All the images were converted into two-dimensional matrix format with area pixel distribution 256*∗*256. To test the recognition model, the selected images were divided into 5 groups in which each group was randomly selected to test the proposed model. Taking the abovementioned sample settings as the base for this experiment, examples of the visual images of martial arts routines are shown in Figure 3.

The article "Artificial Intelligence Auxiliary Algorithm for Wushu Routine Competition Decision Based on Feature Fusion" was retracted in 2023. Reasons: signs of a paper mill; suspected computer-generated content; unreliable results or conclusions; concerns about the data.

### 4.3. Experimental Results

#### 4.3.1. Feature Visualization

We confirmed the feature extraction ability of CNN Wushu routine action recognition through feature visualization. Taking the visual image of Wushu routine action in Figures 2(a) and 2(b) as the test sample, the edge feature segmentation method is used to express the visual feature of Wushu routine action. The result of feature extraction is shown in Figure 4. It is evident that after the application of different filters of CNN, the prominent patterns of CNN are highlighted which can be seen in Figures 4(a) and 4(b).

#### 4.3.2. Recognition Performance

Table 2 summarizes the different recognition results of different feature extraction methods obtained with different classifiers. To further verify the effectiveness of the proposed model, the classification accuracy of different feature extractions methods for visual recognition of martial arts routine movements are verified using the different number of CNN epochs. Table 2 shows that the highest accuracy of 93.98% was achieved by the proposed feature extraction method for 500 epochs whereas the lowest accuracy of 87.15% was obtained by untuned CNN for the same number of epochs. It is also evident that increasing the number of epochs creates a significant effect on the recognition performance of the classification algorithms. It proves the effectiveness and superiority of the algorithm presented in this paper.

#### 4.3.3. Optimization of the Model

The activation function is usually used to perform a nonlinear transformation on the output of the hidden layer of deep neural networks to improve the nonlinear expression ability of the whole network model. For several common activation functions, the ReLU function does not have the problem of gradient disappearance compared with the sigmoid function and tanh function, and its calculation is very simple. Therefore, most CNN adopts ReLU as the activation function. However, the way that the ReLU function directly takes zero on the negative interval makes it easy to transmit the zero gradients back in the process of backpropagation training, resulting in the weight not being updated, that is, the phenomenon of “neuron death” occurs. To solve this problem, ReLU's modified Leaky ReLU function multiplies the value of the negative interval by a very small coefficient *α* to avoid zero gradients. The model convergence effect is shown in Figure 5.

The article "Artificial Intelligence Auxiliary Algorithm for Wushu Routine Competition Decision Based on Feature Fusion" was retracted in 2023. Reasons: signs of a paper mill; suspected computer-generated content; unreliable results or conclusions; concerns about the data.

As can be seen from Figure 5, the performance of ReLU and proposed Leaky ReLU was similar, and both converged the model quickly within the first 150 iterations. The convergence rate of the model using Leaky ReLU was slightly faster because Leaky ReLU solved the problem of neurons not learning when regular ReLU entered a negative range, indirectly increasing the activity of neurons and thus speeding up the convergence rate of the model.

## 5. Conclusion

Competitive Wushu is emerging as a product of the times and is also the artistic carrier of traditional culture China times, and competitive Wushu is a kind of performing arts, through a creative and routine performer to organize routine stylized martial arts action. This paper proposed an artificial intelligence auxiliary algorithm for martial arts routine competition decision-making based on feature fusion. We combined frame segment scanning technology to sample martial arts routine movement visual images and developed a Wushu routine movement feature extraction model. The proposed model achieved the highest recognition accuracy of 93.98% as compared to other feature extraction methods based on deep learning algorithms. The proposed model was evaluated to demonstrate the superior performance of the method in improving the decision-making and action effectiveness instruction ability of Wushu routine competition. In the future, we are planning to incorporate and compare other machine learning algorithms such as RNN and BNN.

## Figures and Tables

**Figure 1:** Video sample of martial arts routine competition.

**Figure 2:** Martial Arts recognition model.

**Figure 3:** Martial arts routines images.

**Figure 4:** CNN feature extraction.

**Figure 5:** Error convergence curve.

**Table 1:** Server configuration.

Class	Parameter
Visual sampling frame frequency	15 kHz
Pixel set of image feature distribution	80
Recognition time interval	2 ms
Area pixel distribution	256*∗*256
Action characteristic decomposition coefficient	0.38, 0.52

**Table 2:** The recognition accuracy of different classifiers.

Accuracy (%)			
Epochs	CNN	LeNet	Proposed
100	85.12	86.51	90.25
200	85.62	88.74	91.27
300	86.14	88.41	92.36
400	86.15	89.25	93.58
500	87.15	89.45	93.98

## Data Availability

The data used to support the findings of this study are included in the article.
